# Breast Cancer Prediction Empowered with Fine-Tuning

**DOI:** 10.1155/2022/5918686

**Published:** 2022-06-09

**Authors:** Muhammad Umar Nasir, Taher M. Ghazal, Muhammad Adnan Khan, Muhammad Zubair, Atta-ur Rahman, Rashad Ahmed, Hussam Al Hamadi, Chan Yeob Yeun

**Affiliations:** ^1^Riphah School of Computing & Innovation, Faculty of Computing, Riphah International University, Lahore Campus, Lahore, 54000, Pakistan; ^2^School of Information Technology, Skyline University College, Sharjah 1797, UAE; ^3^Network and Communication Technology Lab, Center for Cyber Security, Faculty of Information Science and Technology, Universiti Kebangsaan Malaysia, Bangi 43600, Malaysia; ^4^Pattern Recognition and Machine Learning Lab, Department of Software, Gachon University, Seongnam, Gyeonggido 13120, Republic of Korea; ^5^Faculty of Computing, Riphah International University, Islamabad 45000, Pakistan; ^6^Department of Computer Science, College of Computer Science and Information Technology, Imam Abdulrahman Bin Faisal University, P.O. Box 1982, Dammam 31441, Saudi Arabia; ^7^ICS Department, King Fahd University of Petroleum and Minerls, Dhahran 31261, Saudi Arabia; ^8^Center for Cyber Physical Systems, Khalifa University, Abu Dhabi 127788, UAE

## Abstract

In the world, in the past recent five years, breast cancer is diagnosed about 7.8 million women's and making it the most widespread cancer, and it is the second major reason for women's death. So, early prevention and diagnosis systems of breast cancer could be more helpful and significant. Neural networks can extract multiple features automatically and perform predictions on breast cancer. There is a need for several labeled images to train neural networks which is a nonconventional method for some types of data images such as breast magnetic resonance imaging (MRI) images. So, there is only one significant solution for this query is to apply fine-tuning in the neural network. In this paper, we proposed a fine-tuning model using AlexNet in the neural network to extract features from breast cancer images for training purposes. So, in the proposed model, we updated the first and last three layers of AlexNet to detect the normal and abnormal regions of breast cancer. The proposed model is more efficient and significant because, during the training and testing process, the proposed model achieves higher accuracy 98.44% and 98.1% of training and testing, respectively. So, this study shows that the use of fine-tuning in the neural network can detect breast cancer using MRI images and train a neural network classifier by feature extraction using the proposed model is faster and more efficient.

## 1. Introduction

Breast cancer is the most prevalent type of cancer in women, accounting for more than 23% of all female cancers globally. One in every eight to nine women in Western nations will get breast cancer at some time in her life [1]. The identification of a breast cancer tumor at an early stage is critical in the therapy procedure. Mammography is an efficient process because it can detect breast cancer in its early before physical symptoms appear. As an aside, screening mammography is the only test that has been proven to reduce breast cancer too far [2]. To decrease the number of negative cases on radiography, a biopsy is suggested for lesions with a likelihood of more than two percent of suspected cancerous tumors and fewer than thirty percent of them being cancer. Magnetic resonance imaging has lately been utilized for the detection of breast cancer to decrease needless biopsies since it has great soft tissue imaging capabilities and is the most precise tool for identifying illnesses of the breast. Furthermore, the breast does not contain potentially harmful radiation. However, interpreting MRI pictures takes a significant amount of effort and skill on the part of the reader. Additionally, the standardized diagnostic MRI routine takes a long time to obtain and [3] comprises hundreds of pictures. In recent years, computer-aided systems for detecting aberrant lesions and determining tissue characterization in medical imaging have been enhanced [3].

Many of the issues with MRI in terms of breast cancer categorization, detection, and segmentation, such as false-positive rates, limits in indicating cancer-related alterations, poor applicability for follow-up therapy, and subjectivity, have been solved by machine learning and deep learning [4–6]. Machine and deep learning techniques are only successful when the training and test data are from the same feature space and have the same frequency [7]. When the pattern changes, the majority of the quantitative data in the algorithms must be rebuilt from the ground up using a newly acquired categorization model [7, 8]. Acquiring the required training data and developing models in medical applications such as breast imaging is difficult [9]. As a result, it is best to reduce the requirement for the work necessary to get training data [8, 9]. In such cases, it would be preferable to fine-tune from one job to the next [10]. Fine-tuning makes it possible to utilize a previously trained model in another domain as a learning target. As a result, it minimizes the requirement for the labor involved in gathering more training data for retraining [11].

Primary contributions of this study to predict the breast cancer using MRI images with fine-tuning techniques empowered with transfer learning, and the proposed model achieved the highest prediction accuracy which is very helpful for the Internet of medical things and health 5.0.

## 2. Literature Review

Previous research has used several machine learning algorithms to identify breast cancer using MRI scans [12]. The most commonly used public MRI datasets are medical images and signals (MIAS) and the digital database for screening mammography, and fivefold cross-validation is widely used to evaluate classifier models. Some research employed standard automatic feature extraction approaches to acquire characteristics, such as the Gabor filter, the fractional Fourier transform, and the gray level cooccurrence matrix, and then classified them using KNN, support vector machine, or another classifier [13, 14]. As classifiers, neural networks were also employed [15, 16]. In addition, several researches used convolutional neural networks to derive features from breast cancer images [17–19]. As for fine-tuning applications, some of these researches applied previously trained convolutional neural networks. However, few earlier studies presented results achieved using simply a convolutional neural network for both character creation and classification in hysterectomies for the diagnosis of breast cancer.

Convolutional neural networks (CNN) are a widely used technique that produces impressive results in medical imaging, such as brain tumor segmentation [20], pancreatic classification on magnetic resonance imaging [21], intimal thickness assessment, and carotid media in computed tomography [22], to decrease diagnostic mistakes and improve breast cancer detection. CNN learns highly illustrative and ranked features from training breast cancer images [23]. Convolutional neural networks have also gained traction for image classification with excellent sensitivity and specificity. Chen Y. [23] used the U-Net CNN model to segment dynamic contrast breast MRI. Carneiro et al. [24] used unregistered MRI scans and split microcalcifications and a large dataset to fit a convolutional neural network previously trained using ImageNet [25]. For breast cancer classification, shallow CNN, AlexNet, and Google Net were employed, and the effect of initializing pretrained networks on the ImageNet dataset was studied. Rasti [26] presented a mixed-set convolutional neural network for benign cancerous differentiation. Mohiyuddin et al. [27] used the YOLOv5 network to predict breast tumor with the help of a publicly available dataset of curated imaging subset of DDSM [28], and they used augmented techniques and split data 60% and 30% of training and validation, respectively, and achieved 96.50% prediction accuracy. Mehmood et al. [29] used a random forest feature selection technique to predict cervical cancer with the help of a sallow neural network and achieved 93.6% prediction accuracy and 0.07111 mean squared error. Abbas et al. [30] used a proposed model of breast cancer detection that utilized an extremely randomized tree and whale optimization algorithm with the help of a publicly dataset available on Kaggle and achieved a 0.99 F1-score and 0.98 recall. Nowadays, there are automated [31] cognitive smart homes health systems based on machine learning algorithms which are very handy to predict different kinds of diseases, also a collaborative healthcare framework [32] for fitness assessment and cognitive health based on various machine learning and deep learning algorithms.

Previous studies precisely focused on ultrasound and mammogram images for early detection of breast cancer using different machine learning and deep learning techniques. Previous studies lacking in to achieve high prediction accuracy based on machine and deep learning algorithms. This study aims to focus on MRI images for the detection of breast cancer using fine-tuning techniques and using a deep learning classification model empowered with transfer learning.

## 3. Fine-Tuning

Fine-tuning, regardless of the quantity of data supplied, is a typical approach to constructing machine learning models [28]. Training a deep model might necessitate a significant quantity of data and processing resources; nevertheless, fine-tuning can assist in addressing this issue. A previously created model may be applied to different scenarios in a variety of contexts via fine-tuning [33]. For example, you may train a model to do one thing, such as to identify cell kinds and then alter it to do something other, like categorize tumors [33]. In vision tasks, fine-tuning is a critical approach. Fine-tuning research has demonstrated that the learned characteristics of exceptionally large picture sets, such as ImageNet, are highly transferable to a variety of image recognition tasks [34, 35]. The frequently used technique is to replace the previously trained model's last layer with a randomly filled one [36]. Following that, only the top layer variables are trained for the new job, while all other parameters remain constant. Because the fixed portion functions as a feature extractor, this methodology may be considered a feature map application [37].

When the data and tasks are comparable to the data and tasks used to train the original model, this technique works well. When there is insufficient data to train a model for the target task, this type of fine-tuning may be the only option to train a model without overfitting because having fewer variables to train decreases the risk of generalization [38]. When new data for training become available, which is uncommon in medical contexts, the transferred parameters can be thawed and the entire network trained. In this scenario, the original values of the factors [39] are transferred. Using a trained model to begin the weights rather than randomly initializing them can provide a solid start for the algorithm and enhance the number of iterations and fine-tuning [39].

## 4. Research Methodology

With the advancement of artificial intelligence (AI), every gap in medical image processing or other fields uses machine learning techniques to analyze and predict the attributes in medical images. Furthermore, deep learning plays a key role in the early detection of medical images with good efficiency. So, deep learning is very helpful for doctors and patients to procure breast cancer in the early stages. There are multiple diagnosing techniques of AI to detect breast cancer, but deep learning is a very effective approach to predict this before time.

The proposed model of breast cancer prediction is empowered with fine-tuning the use of breast MRI scans for early prediction and procuring the disease in its early stages using different kinds of deep learning approaches. So, the proposed model consists of a training layer and a testing layer. The training dataset consists of breast MRI scans. So, in preprocessing section, all input images from the hospital dataset are converted into 227*∗*227 dimensions for the AlexNet image input layer, and in the training model section, the proposed model imports the pretrained AlexNet model and modifies this model to our desired requirements using fine-tuning. The training model will be stored in the cloud after it achieved the performance measure accuracy; otherwise, the model will retrain and export to the online cloud. During the testing layer, breast MRI scans are acquired as a input and pass into the trained model from intelligent prediction purposes. If the trained model predicts it as “sick,” then we recommend to go to a doctor for consultation, otherwise the patient may go home. So, the detailed proposed model is shown in Figure 1.

## 5. Dataset

The breast MRI scans dataset get from Kaggle which is publicly available for everyone [40]. This breast cancer dataset consists of breast MRI scans of two classes: one is sick and the other is healthy breasts. So, the proposed model uses this dataset for training and testing purposes. A detailed description of the dataset is stated in Table 1, and a sample of sick and healthy breasts is shown in Figure 2.

## 6. Modified AlexNet

At the current time, deep learning approaches are very popular in medical image disease diagnosing with the help of various pretrained algorithms for diagnosing. So, in this paper, we used a pretrained deep learning network of AlexNet for fine-tuning to predict breast cancer with the help of breast MRI scans. So, AlexNet is a pretrained model of CNN, using a pretrained model is known as fine-tuning, and this technique of deep learning is very popular for the prediction of medical diseases. AlexNet algorithm is pretrained using 1000 classes and about 1.5 crore ImageNet datasets. So, we modified AlexNet according to our prediction and class requirements. Modified AlexNet network consists of 5 convolutional with the combination of 5 max pool layers with 3 fully connected layers. Every layer has a combination of activation functions of ReLU. So, the input layer reads images after preprocessing because preprocessing of images is a primary step to getting a proper input stream, and this step can be done with various approaches. In preprocessing, image resizing is a key step to start the AlexNet training process, and images were resized according to AlexNet input layers into 227*∗*227*∗*2, where 2 is for grayscale images and 227*∗*277 are for height and width of images.  Figure 3 shows the sample preprocessed images of breast MRI scans.

So, the last three layers of AlexNet are changed according to our research requirement. The modified AlexNet model is shown in Figure 4.

The last 3 layers of AlexNet were modified according to output class and their labels. Input attributes are fully connected layers for all binary classes. The output size of fully connected (FC) layers is equal to the total label's length. The SoftMax layer is used on the input layer to detect the edge detection which is represented by the convolutional layer while the class features are learned by the FC layer. The convolutional layer is used to extract the features from images by using different filters and preserve the connection between image pixels. So, these FC layers are modified according to our output/prediction class. So, the proposed model of modified AlexNet is trained on binary class labels for the prediction of breast cancer using an MRI scan.

## 7. Simulation and Results

In this research, the article proposed a model that used pretrained AlexNet for the detection of breast cancer before any major consequences. MATLAB 2020a is used for detection purposes. So, the proposed model of breast cancer detection divided the dataset into two parts: the first is training 70% of the data, and the second is testing 30% of the data. So, various statistical performance parameters are used to evaluate the performance of the breast cancer prediction proposed model (e.g., classification accuracy (CA), classification miss rate (CMR), sensitivity, specificity, *F*1-score, positive predicted value (PPV), negative predicted value (NPV), false-positive ratio (FPR), false-negative ratio (FNR), likelihood positive ratio (LPR), and likelihood negative ratio (LNR)). All these statistical performance parameters are used to evaluate the performance of the proposed model. In the proposed model results, á represents true positive results, ß represents true negative results, õ represents false-positive results, and Ø represents false-negative results.

(1) $$\begin{array}{c} \text{CA}=\frac{\text{á}+\beta }{\text{á}+\beta +\delta +\text{Ø}}*100\text{,}\\ \text{CMR}=100-\frac{\text{á}+\beta }{\text{á}+\beta +\text{õ}+\text{Ø}}*100,\\ \text{Sensitivity}=\frac{\text{á}}{\text{á}+\text{Ø}}*100,\\ \text{Specifity}=\frac{\beta }{\beta +\delta }*100,\\ \text{F}1-\text{score}=\frac{2\text{á}}{2\text{á}+\delta +\text{Ø}}*100,\\ \text{F}1-\text{score}=\frac{\text{á}}{\text{á}+\delta }*100,\\ \text{NPV}=\frac{\beta }{\beta +\text{Ø}}*100,\\ \text{FPR}=100-\frac{\beta }{\beta +\delta }*100,\\ \text{FNR}=100-\frac{\text{á}}{\text{á}+\text{Ø}}*100\text{,}\\ \text{LPR}=\frac{\left(\text{á}/\text{á}+\text{Ø}\right)*100}{100*-*\left(\beta /\beta +\delta \right)*100},\\ \text{LNR}=\frac{100-\left(\text{á}/\text{á}+\text{Ø}\right)*100}{\left(\beta /\beta +\delta \right)*100}. \end{array}$$

The proposed model classifies breast cancer in binary classes: one is sick and the second is healthy.  Table 2 shows that breast image data were trained on different epochs using the same learning rate of 0.002, and the best accuracy of the trained model was 98.44% achieved on 10 epochs. The proposed model tried multiple epochs to get optimal results.

Table 3 shows the results of each proposed model's epoch's accuracy, iterations, basic learning rate, and time elapsed. The accuracies are 91.2%, 95.6%, 98.44% of 1 epoch, 5 epochs, and 10 epochs on 10, 50, and 100 iterations, respectively. The proposed model of breast cancer training simulation was improved gradually on different epochs, so the proposed model achieved 98.44% accuracy on 10 epochs and 100 iterations.

Figure 5 shows the sick and healthy images which are generated from the proposed model. It observed that 35 images were labeled as healthy breast and 1 labeled as sick breast.

Table 4 shows the test results of the proposed modern breast cancer detection. There are a total of 420 sample images for testing. From 420 images, 210 images were used to test sick breasts, and 210 images were used for healthy breasts. So, the proposed model predicted 208 healthy breasts, 204 sick breasts, and 6 and 4 images of false positive and false negative, respectively. The healthy class achieved 208 correct images, and the sick class achieved 204 correct images.

Figure 6 shows the training progress of the proposed model on 10 epochs, and the model achieved 98.44% of training accuracy and a 1.66% of loss rate.

Table 5 shows the performance of the proposed AlexNet-based model with respect to different statistical parameters such as accuracy, sensitivity, and specificity during the testing phase. It is observed that proposed model achieved 98.1%, 1.9%, 99%, 97.1%, 98.1%, 97.1%, 99%, 2.9%, 1%, 34.13%, and 0.010% of accuracy, MCR, sensitivity, specificity, *F*1-score, PPV, NPV, FPR, FNR, LPR, and LNR, respectively.

## 8. Conclusion and Future Work

In this study, a breast cancer prediction empowered with the fine-tuning model was used to detect sick and healthy breasts from cancer using MRI images. The statistical performance parameters such as accuracy, miss-classification rate, sensitivity, specificity, *F*1-score, positive predicted value, negative predicted value, false-positive ratio, false-negative ratio, likelihood positive ratio, and likelihood negative ratio state the proposed model achieved the optimal and promising results. So, the proposed model achieves 98.1% and 1.9% of classification accuracy and loss rate, respectively. So, this proposed model can be used in the medical field to prevent unnecessary biopsies and treatment. In the future, this study can be extended by fusing different datasets and applying the fuzzed machine learning concept to the data to get more accurate and promising results.

## Figures and Tables

**Figure 1:** Proposed model of breast cancer prediction using fine-tuning.

**Figure 2:** Sick and healthy breast data samples.

**Figure 3:** Preprocessed (227*∗*227) breast MRI scans.

**Figure 4:** Modified AlexNet model.

**Figure 5:** Classification of images by proposed model of breast cancer detection empowered with fine-tuning.

**Figure 6:** Training progress of proposed model.

**Table 1:** Breast MRI scans dataset detail [40].

Breast cancer state	No. of images
Sick	700
Healthy	700

**Table 2:** Training simulation parameters of the proposed model.

No. of epochs	Learning rate (LR)	No. of layers	Size of images	Pooling method	Mini batch loss
1	0.002	25	227*∗*227*∗*2	MAX	7.8600
5	0.002	25	227*∗*227*∗*2	MAX	1.1209
10	0.002	25	227*∗*227*∗*2	MAX	0.2491

**Table 3:** Performance analysis of proposed model during training.

No. of epochs	Learning rate (LR)	Accuracy (%)	Loss rate (%)	Iterations	Time elapsed (hh:mm:ss)
1	0.002	91.2	8.8	10	00:00:02
5	0.002	95.6	4.4	50	00:00:06
10	0.002	98.44	1.66	100	00:00:11

**Table 4:** Testing confusion matrix of proposed model.

Attributes (420)	Healthy	Sick
Healthy	208	6
Sick	2	204

**Table 5:** Statistical parameter analysis of proposed model during testing.

Instances (420)	Testing (%)
Accuracy	98.1
MCR	1.9
Sensitivity	99
Specificity	97.1
*F*1-score	98.1
PPV	97.1
NPV	99
FPR	2.9
FNR	1
LPR	34.13
LNR	0.010

## Data Availability

The data used in this paper can be requested from the corresponding author upon request.

## References

[1] Berg W. A. (2010). Benefits of screening mammography. *JAMA*.

[2] Fonseca P., Mendoza J., Wainer J., Ferrer J., Pinto J., Castaneda B. (2015). Automatic breast density classification using a convolutional neural network architecture search procedure. *SPIE Proceedings*.

[3] Gitty M., Arabkherademand A., Taheri E. (2017). Magnetic resonance imaging features of adenosis in the breast. *Journal of Breast Cancer*.

[4] Huang Q., Zhang F., Li X. (2018). Machine Learning in ultrasound computer-aided diagnostic systems: a survey. *BioMed Research International*.

[5] Sloun R. J. G. V., Cohen R., Eldar Y. C. (2020). Deep learning in ultrasound imaging. *Proceedings of the IEEE*.

[6] Pan S. J., Yang Q. (2010). A survey on transfer learning. *IEEE Transactions on Knowledge and Data Engineering*.

[7] Brattain L. J., Telfer B. A., Dhyani M., Grajo J. R., Samir A. E. (2018). Machine learning for medical ultrasound: status, methods, and future opportunities. *Abdominal Radiology*.

[8] Khoshdel V., Ashraf A., LoVetri J. (2019). Enhancement of multimodal microwave-ultrasound breast imaging using a deep-learning technique. *Sensors*.

[9] Day O., Khoshgoftaar T. M. (2017). A survey on heterogeneous transfer learning. *Journal of Big Data*.

[10] Weiss K., Khoshgoftaar T. M. (2016). A survey of fine tuning. *Journal of Big Data*.

[11] Ganessan K., Acharya U. R., Chua C. K., Min L. C., Abraham K. T., Ng K. H. (2013). Computer-aided breast cancer detection using mammograms. *IEEE Reviews in Biomedical Engineering*.

[12] Khan S., Hussain M., Aboalsamh H., Bebis G. (2017). A comparison of different Gabor feature extraction approaches for mass classification in mammography. *Multimedia Tools and Applications*.

[13] Narváez F., Alvarez J., Garcia-Arteaga J. D., Tarquino J., Romero E. (2017). Characterizing architectural distortion in mammograms by linear saliency. *Journal of Medical Systems*.

[14] Wang S., Rao R. V., Chen P., Zhang Y., Liu A., Wei L. (2017). Abnormal breast detection in mammogram images by feed-forward neural network trained by jaya algorithm. *Fundamenta Informaticae*.

[15] Nithya R., Santhi B. (2011). Classification of normal and abnormal patterns in digital mammograms for diagnosis of breast cancer. *International Journal of Computer Application*.

[16] Zhu W., Lou Q., Vang Y. S., Xie X. (2017). Deep multi-instance networks with sparse label assignment for whole mammogram classification. *Medical Image Computing and Computer Assisted Intervention − MICCAI 2017*.

[17] Jiao Z., Gao X., Wang Y., Li J. (2016). A deep feature based framework for breast masses classification. *Neurocomputing*.

[18] Dhungel N., Carneiro G., Bradley A. P. The automated learning of deep features for breast mass classification from mammograms.

[19] Havaei M., Davy A., Warde-Farley D. (2017). Brain tumor segmentation with deep neural networks. *Medical Image Analysis*.

[20] Roth H. R., Farag A., Lu L., Turkbey E. B., Summers R. M. (2015). Deep convolutional networks for pancreas segmentation in ct imaging. *SPIE Proceedings*.

[21] Shin J., Tajbakhsh N., Hurst R. T., Kendall C. B., Liang J. Automating carotid intima-media thickness video interpretation with convolutional neural networks.

[22] Hoo-Chang S., Rooth H. R., Gao M. (2016). Deep convolutional neural networks for computer-aided detection cnn architectures, dataset characteristics and fine tuning. *IEEE Transactions on Medical Imaging*.

[23] Chen Y., Xu X., Larsson R. Breast region segmentation being convolutional neural network in dynamic contrast-enhanced mri.

[24] Carneiro G., Nascimento J., Bradley A. P. Unregistered multiview mammogram analysis with pre-trained deep learning models.

[25] Levy D., Jain A. Breast mass classification from mammograms using deep convolutional neural networks.

[26] Rasti R., Teshnehlab M., Phung S. L., Phung S. L. (2017). Breast cancer diagnosis in dce-mri using mixture ensemble of convolutional neural networks. *Pattern Recognition*.

[27] Mohiyuddin A., Basharat A., Ghani U. (2022). Breast tumor detection and classification in mammogram images using modified yolov5 network. *Computational and Mathematical Methods in Medicine*.

[28] (2021). Fine tuning. http://www.isikdogan.com/blog/transfer-learning.html.

[29] Mehmood M., Rizwan M., Gregus M., Abbas S. (2021). Machine learning assisted cervical cancer detection. *Frontiers in Public Health*.

[30] Abbas S., Jalil Z., Javed A. R. (2021). BCD-WERT: a novel approach for breast cancer detection using whale optimization based efficient features and extremely randomized tree algorithm. *Peer J Computer Science*.

[31] Javed A. R., Fahad L. G., Farhan A. A. (2021). Automated cognitive health assessment in smart homes using machine learning. *Sustainable Cities and Society*.

[32] Javed A. R., Sarwar M. U., Beg M. O., Asim M., Baker T., Tawfik H. (2020). A collaborative healthcare framework for shared healthcare plan with ambient intelligence. *Human-centric Computing and Information Sciences*.

[33] Chu B., Madhavan V., Beijbom O., Hoffman J., Darrell T. Best practices for fine-tuning visual classifiers to new domains.

[34] (2021). Convolutional Neural Network Recognition. https://cs231n.github.io/transfer-learning.

[35] Yosinski J., Clune J., Bengio Y., Lipson H. (2014). How transferable are features in deep neural networks?. *Advances in Neural Information Processing*.

[36] Huh M.-Y., Agarwal P., Efros A. A. (2016). What makes ImageNet good for fine tuning?. https://arxiv.org/abs/1608.08614.

[37] Li Z., Hoiem D. (2018). Learning without forgetting. *IEEE Transactions on Pattern Analysis and Machine Intelligence*.

[38] kdnuggets (2021). Building trustworthy and tthical ai systems. https://www.kdnuggets.com/2019/06/5-ways-lack-data-machine-learning.html.

[39] tensorflow (2021). Overfit and underfit. https://www.tensorflow.org/tutorials/keras/overfit_and_underfit.

[40] Kaggle (2021). Breast cancer patients mris. https://www.kaggle.com/uzairkhan45/breast-cancer-patients-mris.

